# Application of an Optical Tracking System for Motor Skill Assessment in Laparoscopic Surgery

**DOI:** 10.1155/2022/2332628

**Published:** 2022-07-22

**Authors:** Lixiao Yang, Kunyong Lyu, Chengli Song

**Affiliations:** ^1^Equipment Department, Shanghai Changhai Hospital, Shanghai 200433, China; ^2^School of Information Science and Technology, Shanghaitech University, Shanghai 201210, China; ^3^Shanghai Institute for Minimally Invasive Therapy, School of Health Science and Engineering, University of Shanghai for Science and Technology, Shanghai 200093, China

## Abstract

**Objective:**

Motion analysis of surgical instruments can be used to evaluate laparoscopic surgical skills, and this study assessed the validity of an optical tracking system for the assessment of laparoscopic surgical motor skills.

**Methods:**

Ten experienced surgeons and ten novices were recruited to complete the transferring tasks on a laparoscopic simulator. An optical tracking system, Micron Tracker, was used to capture the marker points on each instrument and to obtain the coordinates of the marker points and the corresponding instrument tip coordinates. The data are processed to create a coordinate system based on the laparoscopic simulator and to calculate the movement parameters of the instruments, such as operating time, path length, speed, acceleration, and smoothness. At the same time, the range of motion of the instrument (insertion depth and pivoting angle) is also calculated.

**Results:**

The position that the tip of the instrument can reach is a small, irregularly shaped spatial area. Significant differences (*p* < 0.05) were found between the surgeon and novice groups in parameters such as operating time, path length, mean speed, mean acceleration, and mean smoothness. The range of insertion depth of the instruments was approximately 150 mm to 240 mm, and the pivoting angles of the left and right instruments were 30.9° and 46.6° up and down and 28.0° and 35.0° left and right, respectively.

**Conclusions:**

The optical tracking system was effective in subjectively evaluating laparoscopic surgical skills, with significant differences between the surgeon and novice groups in terms of movement parameters, but not in terms of range of motion.

## 1. Introduction

Laparoscopic surgery is the quintessential example of minimally invasive surgery [1, 2], which is routinely performed through multiple (3-5) tiny (5-12 mm) incisions and has a wide range of clinical applications. Due to the use of rigid slender instruments, the lack of tactile feedback, the fulcrum effect, and the lack of a sense of depth, surgeons require a higher level of skill in laparoscopic manipulation compared to conventional open surgery. One of the objective indicators for evaluating surgical skills is the movement parameters of the instruments [3–6], and when the operator is skilled at a particular task, he/she will demonstrate more effective instrument movements, as reflected in the movement parameters of the instruments.

The measurement of motion parameters of instruments has been achieved by various methods [7–10], such as electromagnetic positioning, mechanical means, and optical tracking. The motion parameters evaluated are usually the path length, speed, acceleration, smoothness of the instrument, etc. These parameters are either path accumulations of the instrument position or derivatives of the different values for the operation time [11–13]. The optical tracking system has many advantages over electromagnetic positioning and mechanical methods. Firstly, it is a noncontact measurement method that does not require much modification to the measurement target, does not require the use of cables to transfer data, and does not require a marker to be placed on the measured target. Secondly, the use of electromagnetic equipment is inevitable in the actual surgical environment, and this inevitably interferes with the electromagnetic positioning system [14–16], whereas the optical capture system is not affected. The disadvantage is that there must not be an obstacle between the marker point to be measured and the optical tracking system to block the propagation of light, which can be solved by the proper design and installation of the marker point.

The main objective of this study was to evaluate the validity of an optical tracking system, the Micron Tracker, for the assessment of motor skills in laparoscopic surgery. Innovatively, the data from two different operating levels (surgeon and novice groups) were tested using the optical tracking system to record the position of the instruments during the operation. The coordinates of key points on the laparoscopic simulator were obtained and used to create a coordinate system from which the motion parameters of the instruments, such as time, path length, speed of movement, acceleration, and smoothness, as well as the range of motion of the instruments (insertion depth and pivoting angle), were calculated. The differences between the surgeon group and the novice group are analyzed.

## 2. Materials and Methods

### 2.1. Experimental Platform

The experimental platform consists of a simulator and an optical tracking system (Figure 1(a)): (1) The simulator is a product of Shanghai Shide Medical Technology Co., Ltd. A built-in camera is used to transmit the image from inside the simulator to the monitor. (2) The optical tracking system uses a third-generation Micron Tracker from Claron Technology Inc. of Canada, camera model H3-60, which captures the 3D coordinates of marker points within its field of view in real time. It is widely used for skills assessment, visual navigation, etc. [13, 17–19]. In this study, two types of markers were designed and fixed to the proximal end of the instrument (Figure 1(b)), which are lightweight and robust enough not to interfere with the normal use of the instrument. The Micron Tracker captures the location of the marker and obtains the position of the instrument tip by calibration. Two 5 mm standard length gripping forceps (Shanghai Shide Medical Technology Co., Ltd., Shanghai) were used for this study.

### 2.2. Task Setting

This study set out to test the “left-right ring transfer” training task, which focuses on the operator's hand-eye coordination and two-handedness [20]. The task requires the trainer to use the left hand to grab the rubber ring from the left post, pass it to the right hand and attach it to the right post. After the 4 rubber rings have been placed on the right post one by one, the process is reversed, with the right hand grabbing the rubber ring and passing it to the left hand and placing it on the left post, in turn, to complete the training. The training task is shown in Figure 2.

### 2.3. Operators

Ten surgeons and ten school students who are right-handed, without any hand disabilities and with a corrected vision of at least 1.0 are recruited as operators for the task. The purpose and content of the training task and the specific task steps are explained to the volunteers before operating. All operators were given 10 minutes to familiarize themselves with the task content. Each operator completed the task three times in succession, and the average of the calculated results was taken as the data for that operator.

### 2.4. Measurement Process

After commissioning the experimental equipment and waiting for the Micron Tracker camera to warm up and stabilize, the measurements are started. The type of marker and the corresponding instrument tip point are registered in the optical tracking system. Each operator repeatedly completes the task three times. Data are recorded including time, the position of the instrument marker point, and the position of the instrument tip. Once the task is completed, the trocar is removed, and the coordinates of the two insertion points are measured using the test tool that comes with the optical tracking system, and the coordinates of the center point of the task board are measured using the surgical instruments. Data processing and analysis are carried out after the completion of all tests.

### 2.5. Data Processing

All data were imported into MATLAB R2015a (MathWorks, Inc., Natick, MA, USA) for analysis to extract the tip point positions of the left and right instruments and the time corresponding to each position. The first step was to create a coordinate system based on the three key points on the laparoscopic simulator, instrument left insertion point *A*, right insertion point *B*, and task board center *C*. Using the midpoint *O* of *A* and *B* as the origin, *O*⟶*B* as the positive direction of the *x*-axis, and *O*⟶*C* as the approximate positive direction of the *z*-axis, a coordinate system based on the laparoscopic simulator was established according to Figure 3 [21].

The measured data such as points reached by the instrument tip and insertion points were then converted to coordinate values in the new coordinate system, and the original data were smoothed using a sliding average filter to smooth the data (*n* = 3). The processed point cloud data of the instrument tip and the key point data were imported into the 3D model of the laparoscopic simulator via Unigraphics (Siemens PLM Software, Plano, TX, USA) software and aligned according to the established coordinate system *Oxyz* to show the position of the instrument relative to the laparoscopic simulator.

Parameters such as path length, speed, acceleration, and smoothness of the instrument are calculated [13]. The definition and calculation of the instrument movement parameters are shown in Table 1. The movement parameters are calculated separately for each operator's left and right-handed instrument.

Finally, the range of motion of the instrument is calculated. The insertion depth of the instrument is the distance from the insertion point to the tip of the instrument, and the pivoting angle of the instrument is the angle between the instrument and the plane of the coordinate system. As shown in Figure 3, the left and right pivoting angles of the instrument concerning the plane *Oyz* and the up and down oscillation angles are the angles of the instrument with respect to the plane *Oxz*.

### 2.6. Statistical Analysis

Based on Table 1, the operating time, path length, average speed, maximum speed, average acceleration, maximum acceleration, average smoothness, and maximum smoothness of the left-hand and right-hand instruments were calculated for each operator. The insertion depth and pivoting angle of the left and right-hand instruments were calculated for each operator based on the calculation of the range of motion of the instruments. A one-way ANOVA was used to investigate the differences between the surgeon and novice groups, with *p* < 0.05 being considered statistically significant. Results are expressed as mean ± standard deviation.

## 3. Results

### 3.1. Trajectory of the Tip of the Instrument

The location of all the tip points of each instrument forms a spatial range, and although the tip points of each operator's instrument are not the same, they are all a small, irregularly shaped set of spatial points. This point set is contained within the theoretical conical space accessible to the instrument (Figure 4).

### 3.2. Instrument Movement Parameters and Range of Motion

The movement parameters and range of motion of the instrument are shown in Table 2. All parameters are divided into left and right instruments, except for the time parameter, and all parameters are greater for the right instrument than for the left instrument.

In terms of movement parameters, the time required to complete the task was shorter for the surgeons than for the novice group (82.1 s vs. 151.4 s, *p* < 0.001) and the distance travelled at the tip of the instrument was smaller (*p* < 0.001), while the mean movement speed, acceleration, and smoothness were significantly greater than for the novice group (*p* < 0.05). On the other hand, there was no significant difference between the surgeon and novice groups in terms of maximum speed, acceleration, and smoothness of the instruments (*p* > 0.05). The maximum speed, acceleration, and smoothness of the instruments held in the right hand (dominant hand) were higher in the novice group than in the surgeon group.

In contrast, there was no significant difference in the range of motion of the surgical instruments within the laparoscopic simulator (*p* > 0.05). The depth of insertion of the instruments was approximately 150 mm to 240 mm, with a range of approximately 90 mm, and the insertion depths of the left and right instruments were similar; the up and down pivoting angles of the instruments were approximate: -19.0° to 11.9° (left instruments) and -24.5° to 22.1° (right instruments), with a range of 30.9° and 46.6°, respectively, with the up and down pivoting angle of the right instruments being significantly higher than that of the left instruments. The left and right pivoting angles of the right instrument are slightly higher than those of the left instrument, with 4.8° to 32.8° (left instrument) and -34.8° to 0.2° (right instrument), with a range of 28° and 35°, respectively.

## 4. Discussion

The measurement of the key points of the laparoscopic simulator is subject to error. As the two groups of researchers in this study were from the hospital and the university, respectively, the experimental set-up was moved several times and the key points had to be remeasured for each change of position. In addition, the trocar and the soft material surrounding it are unstable in practice, and the rotation points of the instruments can drift. The insertion point and the center of the task plate are the basis for establishing the coordinate system, and therefore, there may be differences between the coordinate systems. When analyzing the results, attention is paid to the upper and lower limits of instrument pivoting along with the magnitude of the pivoting. In this study, only the interval size (maximum minus minimum) was considered when statistically analyzing the range of motion of the instrument.

In a previous study of the range of motion of laparoscopic instruments, the author hypothesized [21]: “The characteristics of instrument movement will vary depending on the operator's operating habits, proficiency of surgical skills, etc. In particular, parameters such as speed, acceleration and smoothness of instrument movement have been used as objective indicators for judging surgical skills. However, the instrument movement space of interest in this paper is influenced by the operating target, and the tip of the instrument will only operate around and in the vicinity of the operating target. Although there will be small differences between operators, the effect on the calculation method and even the movement space itself is minimal.” This study grouped operators according to their skill level, and the results of the calculations fully support this hypothesis.

The data in Table 2 show that the movement parameters calculated by the optical tracking system were able to distinguish between the surgeon and novice groups, demonstrating the validity of the optical tracking system in evaluating motor skills in laparoscopic surgery. The result is generally consistent with other evaluations of optical tracking systems [13].

There were significant differences in the movement parameters between the surgeon and novice groups, with the surgeon taking less time to complete the task and moving the instrument a smaller distance, while the average movement speed, acceleration, and smoothness were significantly greater than in the novice group, indicating that the surgeon operated the instrument with better economy and that the surgeon operated it significantly more effective than the novice group, using less time and less distance to complete the same task. In terms of parameters such as maximum speed, acceleration, and smoothness, although there were no significant differences between the two groups, for instruments held by the right hand (dominant hand), the maximum speed, acceleration, and smoothness were higher in the novice group than in the surgeon group. These parameters reflect, to some extent, the abrupt changes (smoothness), the forces (acceleration), etc., during the manipulation of the instruments. The instruments operated by the dominant hand move more frequently and too abrupt changes may cause damage to human tissues during surgical operations, indicating that the novice group is less able to control the instruments than the surgeon group.

The range of motion of the instruments does not vary significantly depending on the level of the operator. The main factors influencing the range of motion of the instruments were the type of task, the position of the insertion point, and the right and left-handedness [18]. The statistics in Table 2 show that the range of motion of right-handed instruments is significantly higher than that of left-handed instruments, both in terms of the depth of insertion of the instrument and the angle of swing in both directions.

On this basis, the study was based on the alignment of the newly constructed coordinate system and the measured instrument tip points were imported into the laparoscopic simulator via the 3D software Unigraphics (Figure 4) to visualize the movement of the instruments within the training box more visually. This can be useful for the analysis of surgical approaches and can also provide ideas for the design of instruments under new surgical approaches.

## 5. Conclusion

In this paper, the optical tracking system Micron Tracker can distinguish between the surgeon and novice groups and the range of motion of the instruments is not influenced by the skill level of the operator. This optical tracking system is a noncontact measurement that is expected to be used in clinical applications.

## Figures and Tables

**Figure 1:** Experimental platform: (a) laparoscopic simulator and optical tracking system and (b) laparoscopic instrument with markers.

**Figure 2:** Ring transfer training tasks.

**Figure 3:** Coordinate system on the laparoscopic simulator.

**Figure 4:** Position of the instrument tip for the simulator.

**Table 1:** Definition and calculation of movement parameters.

Parameters	Definition	Calculation method
Time (s)	Time to complete the task	*T* = *t*_*f*_ − *t*_0_
Length of the path (mm)	Distance to be travelled to complete the tip of the mission apparatus	$L_{i}=\sqrt{{\left({dr}_{xi}\right)}^{2}+{\left({dr}_{yi}\right)}^{2}+{\left({dr}_{zi}\right)}^{2}}$
Speed (mm/s)	Change in position of the tip of the instrument relative to time	$v_{i}=\sqrt{{\left({dr}_{xi}/dt\right)}^{2}+{\left({dr}_{yi}/dt\right)}^{2}+{\left({dr}_{zi}/dt\right)}^{2}}$
Acceleration (mm/s^2^)	Variation of the velocity of the tip of the instrument relative to time	$a_{i}=\sqrt{{\left({dv}_{xi}/dt\right)}^{2}+{\left({dv}_{yi}/dt\right)}^{2}+{\left({dv}_{zi}/dt\right)}^{2}}$
Smoothness (mm/s^3^)	Variation of instrument tip acceleration concerning time	$j_{i}=\sqrt{{\left({da}_{xi}/dt\right)}^{2}+{\left({da}_{yi}/dt\right)}^{2}+{\left({da}_{zi}/dt\right)}^{2}}$

**Table 2:** Comparison of the movement parameters of the instruments in the transferring task between the surgeon and novice groups.

	Surgeon group	Novice group	*p* value
Operating time (s)	82.1 ± 12.6	151.4 ± 18.8	0.000^∗^
Distance travelled by left instrument (mm)	1703.8 ± 17.9	2675.2 ± 34.0	0.000^∗^
Distance travelled by right instrument (mm)	1866.9 ± 11.3	2573.3 ± 39.0	0.000^∗^
Maximum speed of left instrument (mm/s)	251.0 ± 87.6	192.9 ± 52.1	0.115
Maximum speed of right instrument (mm/s)	310.0 ± 47.2	331.4 ± 111.2	0.664
Average speed of left instrument (mm/s)	38.0 ± 5.6	32.2 ± 4.3	0.035^∗^
Average speed of right instrument (mm/s)	48.3 ± 3.9	38.8 ± 4.3	0.001^∗^
Maximum acceleration of the left instrument (mm/s^2^)	1702.3 ± 645.1	1432.7 ± 411.7	0.321
Maximum acceleration of the right instrument (mm/s^2^)	2081.8 ± 339.5	2217.1 ± 693.8	0.665
Average acceleration of left instruments (mm/s^2^)	262.4 ± 41.6	223.0 ± 22.9	0.027^∗^
Average acceleration of the right instrument (mm/s^2^)	343.8 ± 31.3	273.4 ± 24.6	0.000^∗^
Maximum smoothness of the left instrument (mm/s^3)	12804.3 ± 4206.2	11447.6 ± 2996.7	0.463
Maximum smoothness of the right instrument (mm/s^3)	15998.2 ± 3456.7	17134.7 ± 4713.0	0.617
Average smoothness of left instrument (mm/s^3)	2137.4 ± 356.6	1824.3 ± 170.3	0.031^∗^
Average smoothness of the right instrument (mm/s^3)	2815.8 ± 278.8	2240.3 ± 187.0	0.000^∗^
Depth of insertion of left instrument (mm)	80.2 ± 10.6	84.4 ± 16.1	0.579
Depth of insertion of right instrument (mm)	84.2 ± 6.7	95.3 ± 19.8	0.210
The angle of rotation of the left instrument around the *x*-axis (°)	34.1 ± 8.4	29.9 ± 4.1	0.196
The angle of rotation of the right instrument about the *x*-axis (°)	46.3 ± 5.7	47.5 ± 10.4	0.794
The angle of rotation of the left instrument around the *y*-axis (°)	28.2 ± 3.9	28.5 ± 5.1	0.692
The angle of rotation of the right instrument around the *y*-axis (°)	33.6 ± 4.9	35.2 ± 8.9	0.707

^∗^ *p* < 0.05, statistically significant.

## Data Availability

The data used to support this study are available from the corresponding author upon request.
